The article "miR-138 Reduces the Dysfunction of T Follicular Helper Cells in Osteosarcoma via the PI3K/Akt/mTOR Pathway by Targeting PDK1" was retracted in 2023. Reasons: signs of a paper mill; suspected computer-generated content; unreliable results or conclusions; concerns about the data.

# miR-138 Reduces the Dysfunction of T Follicular Helper Cells in Osteosarcoma via the PI3K/Akt/mTOR Pathway by Targeting PDK1

**DOI:** 10.1155/2021/2895893

**Published:** 2021-12-14

**Authors:** Baoen Jiang, Xiuqin Kang, Gang Zhao, Jianshu Lu, Zhitao Wang

**Affiliations:** ^1^Department of Traumatic Orthopaedics, Dongying People's Hospital, No. 317 Nanyi Road, Dongying District, Dongying, Shandong 257091, China; ^2^Department of Nursing, Dongying People's Hospital, No. 317 Nanyi Road, Dongying District, Dongying, Shandong 257091, China

## Abstract

**Objective:**

To study the effect of miR-138 on the function of osteosarcoma (OS) T follicular helper cells (Tfh cells) and its mechanism.

**Methods:**

Peripheral blood mononuclear cells (PBMCs) were isolated from patients with osteosarcoma (OS group) and healthy volunteers (control group). CD4+CXCR5+ Tfh cells and CD9+ B cells were sorted by flow cytometry. qRT-PCR was used to detect the expression of miR-138 and PDK1 in the peripheral blood and CD4+CXCR5+ Tfh cells. Flow cytometry was employed to detect the proportion of CD4+CXCR5+ Tfh cells in CD4+ T cells, the level of CD40L in CD4+CXCR5+ Tfh cells, and the expression of CD27 and CD38 in B cells. Western blot was used to determine the protein expression of PDK1, PI3K, p-Akt, Akt, p-mTOR, and mTOR. In addition, dual-luciferase reporter assay was performed to verify the relationship between miR-138 and PDK1. ELISA method was used to determine the levels of IgM, IgG, IL-10, and IL-21.

**Results:**

Compared with that of the control group, the expression of miR-138 in PBMC and CD4+CXCR5+ Tfh cells of the OS group was lower; overexpression of miR-138 could promote the maturation of Tfh cells and immature B cells. The results of the dual-luciferase report experiment showed that miR-138 can target and negatively regulate PDK1, and PDK1 can reverse the effect of miR-138 on the function of Tfh cells and immature B cells.

**Conclusion:**

miR-138 inhibits the PI3K/Akt/mTOR pathway by targeting and negatively regulating PDK1 to alleviate the dysfunction of T follicular helper cells in OS.

## 1. Introduction

Osteosarcoma (OS) is the most common primary malignant bone tumor in adolescents, and it is also the most difficult-to-treat tumor in orthopedics [1]. According to the statistics of our country (China), the incidence of OS ranks the first among primary malignant bone tumors, accounting for 15% of all primary bone tumors [2], with a high degree of malignancy and extremely poor prognosis. It can metastasize to the lung within few months [3], and its survival rate of 3-5 years after amputation is only about 60%. Although there has been some progress in the etiology, development, diagnosis, and treatment of OS in recent years, the specific pathogenesis is still unclear. At the same time, it lacks effective targets for the diagnosis and treatment of OS.

MicroRNAs (miRNAs) are small single-stranded RNAs about 21-25 nt that do not code proteins. Its expression changes are related to the occurrence, development, diagnosis, and prognosis of the tumor [4]. It is worth noting that miRNAs have an important characteristic, that is, they are very stable in plasma and serum and will not be degraded by RNase [5]. To find miRNA biomarkers with specific expression patterns will be of great significance for OS early diagnosis and treatment.

miR-138 has been reported as a tumor suppressor gene with low expression in different malignant tumors [6–8]. Studies have reported that miR-138 is lowly expressed in OS, and overexpressing of miR-138 can inhibit the proliferation and invasion of OS cells and promote apoptosis by suppressing DEC2 expression [9]. Meanwhile, miRNA-138-5p can be used as a biomarker for poorer prognosis in children, adolescents, and young adults with OS [10]. In recent years, studies have shown that miR-138 has tumor immunomodulatory effects. For example, miR-138 treatment of GL261 glioma in immune-competent mice showed significant regression, the median survival time of mice increased by 43% (*P* = 0.011), and the expression of FoxP3+ regulatory T cells was reduced. However, this therapeutic effect has been lost in nude mice with poor immunity and lack of CD4+ or CD8+ T cells, and direct treatment of miR-138 at physiological did not inhibit the growth of glioma cells [11]. In oral squamous cell carcinoma (OSCC), preimmunization with miR-138-rich *γδ*TDEs can inhibit the development of OSCC in immunocompetent C3H mice, but has no effect on nude mice, suggesting that miR-138-rich *γδ*TDEs have immunomodulatory effects [12]. These results confirm that miR-138 may exert its anticancer effects by regulating T cell function. However, the effect of miR-138 on T cells in patients with OS is unclear.

T follicular helper cells (Tfh) are currently a research hotspot in basic immunology. Originally reported by Schaerli et al. [13] in 2000, Tfh cells were differentiated from primitive Th cells under the action of their specific transcription factor B cell lymphoma factor-6 (Bcl-6) [14], continued to highly express the surface molecule CXCR5 and release the cytokines of IL-10, IL-6, and IL-21. After IL-21 and B cells meeting each other at the lymphoid follicles and combining with their IL-21 receptors, they promoted the proliferation and differentiation of B cells in large numbers and secreted IgM, IgG, IgA, and other antibodies [15]. Meanwhile, it will produce memory B cells and plasma cells and further assisted the conversion of immunoglobulin. The functional detection of Tfh cells and the verification of their interaction with B cells are important breakthroughs in humoral immunity. The study by Guo et al. [16] found that patients with non-small-cell lung cancer (NSCLC) have a significantly higher proportion of circulating Tfh cells than normal people. Hollern et al. [17] further confirmed that immune checkpoint therapy can exert antitumor efficacy by inducing Tfh to activate B cells. These findings indicated that Tfh cells are critical in tumor immunotherapy. OS has obvious inherent instability and high immunogenicity, and the antitumor immune response is ineffective for OS. Gao et al. [18] suggest that this may be due to impaired of IL-21 secretion capacity in Tfh cells in OS. He et al. [19] found a significant abundance of Tfh cells and CD8+ T cells in OS patients with good immune response by immune infiltration analysis. These studies suggest that Tfh is involved in the immune regulation of OS. However, there is no research on the effect and mechanism of miR-138 on Tfh cells in OS. Therefore, in this study, we first determined the expression of miR-138 in OS and Tfh cells and further explored its effect on Tfh cell function and mechanism by interfering with miR-138 expression, in order to provide a basis for clinical immunotherapy of OS.

## 2. Methods

### 2.1. Research Object

15 cases of patients with OS (OS group) diagnosed by postoperative histopathological analysis and 15 cases of healthy volunteers (control group) who underwent physical examination were collected in Dongying People's Hospital. Among them, 8 were males and 7 were females, aged from 20 to 50 years old. All participants provided informed consent, and this study was approved by the ethics committee of Dongying People's Hospital.

### 2.2. Serum Collection and Isolation and Culture of the Peripheral Blood Mononuclear Cells (PBMCs)

4 ml of fasting blood from OS patients and healthy controls was collected and placed in sodium citrate anticoagulant blood vessels to centrifuge, and the supernatant was following the instructions of the human whole blood mononuclear cell separation solution (Solarbio, China) and gradient centrifugation to obtain PBMCs. The anticoagulant pellet was added into PBS. The blood cells mixed with PBS were slowly added to the surface of the lymphocyte separation liquid, and the ratio of the diluted blood to the separation liquid was 2 : 1. Then, after centrifuging at 1500 rpm for 20 min, the liquid was divided into three layers, from top to bottom was plasma (light yellow), white blood cell layer (milk white), and blood cell layer (red). We collected the white blood cell layer with a Pasteur pipette, centrifuged the tube at 10000 rpm for 5 min, then discarded the supernatant, resuspended the cells, added 10% fetal bovine serum (FBS) and 1% penicillin-streptomycin RPMI 1640 medium, and finally cultured it in an incubator at 37°C and 5% CO_2_.

### 2.3. qRT-PCR

TRIZOL (Invitrogen, Carlsbad, CA, USA) was used to extract total RNA, which were reversely transfected into the cDNA by the reverse transcription kit (TaKaRa, Tokyo, Japan). The PCR reaction was carried out following the instructions of the Fluorescence Quantitative PCR Kit (SYBR Green Mix, Roche Diagnostics, Indianapolis, IN). The thermal cycling parameters were 95°C for 10 s, then 95°C for 5 s, 60°C for 10 s, 72°C for 10 s, a total of 40 cycles, and the last extension at 72°C for 5 min. There were 3 replicates for each quantitative PCR. GAPDH and U6 were selected as internal references. The experimental data were analyzed by the 2^-*ΔΔ*Ct^ method. The primer sequences of genes and their internal references are shown in Table 1.

### 2.4. Tfh Cell Sorting

We resuspended each 107 PBMC with 40 *μ*l magnetic-activated cell sorting (MACS) buffer and added 10 *μ*l CD4+ T cell Biotin-Antibody Cocktail. After incubating at 4°C in the dark for 5 min, we added 1 ml MACS buffer to wash, centrifuged at 1500 r/min for 5 min, and discarded the supernatant. After resuspending the cells in 30 *μ*l MACS buffer, 20 *μ*l CD4+ T cell Microbead Cocktail was added and incubated at 4°C in the dark for 10 min, and then, 1 ml MACS buffer was added for washing, centrifuged at 1500 r/min for 5 min, and discarded the supernatant. Later, the sorting column-MS column, magnet block, and magnetic stand were placed out, the column was moistened with 500 *μ*l MACS buffer, and the cells were resuspended in 500 *μ*l MACS buffer. The cell suspension was passed through the column to collect the effluent, and then, the column was washed 3 times with 500 *μ*l MACS buffer to further collect the effluent. Finally, we collected all the cell suspension obtained 4 times, centrifuged it at 1500 r/min for 5 min, and discarded the supernatant, and the cells left were CD4+ T cells.

FITC-CD4/APC-CXCR5 antibody was used to label CD4+CXCR5+ Tfh cells. CD4+ T cells obtained above were added with FITC-CD4, APC-55-CXCR5 antibody (BD Bioscience, USA), incubated at 4°C in the dark for 30 min. Then, 1 ml FACS buffer was added for washing and centrifuged at 1500 r/min for 5 min, and the supernatant was discarded. And then, the cells were resuspended with 200 *μ*l FACS buffer and transferred to a sterile flow cytometer. We later turned on the FACSAria flow cytometer (BD, USA), adjusted it to the best working conditions, and chose both CD4 and CXCR5 positive to sorting. The collection solution was PBS containing 30% FCS, and 10^6^ cells were collected within about 20 min. Part of the collected liquid was remained to test the purity of Tfh cell sorting, some cells were subjected to qRT-PCR and Western blot to detect the expression of miR-138 and PDK1, and the remaining cells were returned to the incubator for culture.

### 2.5. B Cell Isolation and Culture

We used CD19 antibody to label B cells, resuspended each 10^7^ PBMC with 90 *μ*l MACS buffer to mix them well, then added 10 *μ*l anti-CD19 microbeads, tapped the bottom of the tube to mix, and then incubated it at 4°C for 15 min in the dark. Then, 1 ml buffer was added to rinse the cells, and then, it was centrifuged at 300 *g* for 10 min; the supernatant was discarded. In the final, 1 ml buffer was added to resuspend the cells and the MidiMACS sorter was employed to sort and collect CD19+ B cells.

### 2.6. Cell Transfection

When the CD4+CXCR5+ Tfh cells isolated from the OS group grew to 50-60% confluence in a plate with 6 wells, we transfected the miR-138 mimics and its negative control (NC mimics), miR-138 inhibitor and its negative control (NC inhibitor), and pcDNA3.1-PDK1 overexpression vector and empty pcDNA3.1 (NC vector, 2 *μ*g) (GenePharma, China) into the cells according to the instructions of Lipofectamine 2000 reagent (Invitrogen, Carlsbad, CA, USA).

### 2.7. Coculture of the CD4+CXCR5+ Tfh Cells and B Cells

The transfected CD4+CXCR5+ Tfh cells and purified B cells were mixed and cultured at a ratio of 3 : 1, and the cell culture supernatant was collected on the seventh day to determine the contents of IgG, IgM, IL-10, and IL-21.

### 2.8. ELISA

After collecting the cell culture supernatant of each group, the concentration of IgM, IgG, IL-10, and IL-21 in the cell culture supernatant was detected using an ELISA kit (R&D, USA). All operations were carried out strictly followed by the ELISA kit instructions.

### 2.9. Dual-Luciferase Reporter Experiment

Through the online database TargetScan (http://www.targetscan.org/vert_72/), we predicted the binding site of miR-138 and PDK1. According to the predicted results, the wild sequence and mutant sequence (wt-PDK1, mut-PDK1) of the binding site were designed and synthesized. The wild sequence and the mutant sequence of the binding site were inserted into the luciferase reporter gene vector (pGL3-Basic) and then cotransfected with miR-138 mimics (GenePharma, China) and NC mimics into 293T cells (Shanghai Cell Bank, Chinese Academy of Sciences). After 48 hours of transfection, the dual-luciferase detection system was used to detect the relative luciferase activity levels between different groups.

### 2.10. Western Blot

RIPA Lysis Solution (Biyuntian, China) was used to lyse cells to obtain protein samples. After determining the protein concentration using the BCA kit (Biyuntian, China), the protein was separated by 10% SDS-PAGE and then transferred to the PVDF membrane. After being blocked in 5% BSA blocking solution for 1 h at room temperature, the membrane was added with the primary antibodies GAPDH (5174S, 1 : 1000), PDK1 (5662S, 1 : 1000), PI3K (4225S, 1 : 1000), Akt (9272S, 1 : 1000), P-Akt (4060S, 1 : 1000), mTOR (2983S, 1 : 1000), and p-mTOR (5536S, 1 : 1000) (Cell Signaling, USA), incubated overnight at 4°C. On the next day, it was incubated with the secondary antibody horseradish peroxidase-labeled goat anti-rabbit IgG (1 : 5000, CWBIO, China) for 1 h at room temperature. After washing the membrane, we added a chemiluminescence developer dropwise, used a chemiluminescence imaging system (Bio-Rad) for detection, and analyzed the gray value of protein bands by ImageJ software.

### 2.11. Statistical Analysis

The data obtained were analyzed and graphed using SPSS 18.0 (IBM Corp., Armonk, NY, USA) and GraphPad Prism 7 (GraphPad Software Inc., USA), respectively. Comparisons between groups used *t*-test or one-way analysis of variance (Dunnett's method), and correlation analysis adopted Pearson analysis. The experimental data are expressed as mean ± standard deviation (SD). All experiments were repeated 3 times, and the difference was significant when *P* < 0.05.

## 3. Results

### 3.1. miR-138 Is Downregulated in PBMC and Tfh Cells of OS Patients

The expression level of miR-138 in the PBMC of OS patients was distinctly lower than that of normal people detected by qRT-PCR (Figure 1(a)). The result of flow cytometry detecting the proportion of CD4+CXCR5+ Tfh cells in the isolated PMSCs showed that the proportion of CD4+CXCR5+ Tfh cells in the CD4+ T cells of the OS group was notably increased (Figures 1(b) and 1(c)). The expression of miR-138 in CD4+CXCR5+ Tfh cells of OS patients was also obviously downregulated, which was consistent with the results of PBMC (Figure 1(d)). Correlation analysis also indicated that the proportion of CD4+CXCR5+ Tfh cells was negatively correlated with the expression of miR-138 (Figure 1(e)). These results suggested that miR-138 may be involved in regulating the immune response of OS.

### 3.2. miR-138 Increases CD40L Level in Tfh Cells and Promotes B Cell Maturation in OS Patients

Mature B cells can produce diverse B cell pools and high-affinity B cell antigen receptors (BCRs) for pathogen removal, while T cells can increase the affinity of B cells and induce the maturation of B cells [20]. The tumor necrosis factor-related activator protein CD40L is expressed in activated CD4+ T lymphocytes and can induce the activation and proliferation of B cells [21], and CD27 and CD38 are the maturation signs of B cells. We first intervened in the expression of miR-138 and used qRT-PCR to verify the transfection efficiency. The results showed that when the Tfh cells of OS patients were transfected with miR-138 mimics, the expression of miR-138 in the cells was notably higher, and when the cells were transfected with miR-138 inhibitor, the expression was lower (Figure 2(a)). Subsequently, when miR-138 was overexpressed in Tfh cells, the proportion of CD40L was higher, and when miR-138 was knocked down, the proportion of CD40L was obviously lower (Figure 2(b)). After further cocultivating Tfh cells with B cells, the proportion of CD27 and CD38 in B cells showed that after cocultivation with Tfh cells overexpressing miR-138, the proportions of CD27 and CD38 in B cells were notably higher, and after knocking down the miR-138, their proportions reduced (Figure 2(c)). At the same time, the levels of IgM, IgG, IL-10, and IL-21 in the supernatant after cocultivation were tested, and the results also showed that their levels were notably higher after overexpressing miR-138 (Figures 2(d)–2(g)), indicating that miR-138 can promote Tfh cells to secrete related cytokines to promote the maturation of B cells.

### 3.3. PI3K/Akt/mTOR Pathway Is Inhibited in Tfh Cells of OS Patients

The PI3K/Akt/mTOR pathway is a common reason in tumorigenesis and development, and its involvement in OS has been reported in the literature. At the same time, it has been reported that miR-138 can inhibit the PI3K/Akt/eNOS pathway [22]. Therefore, we speculated whether miR-138 also affects the PI3K/Akt pathway in OS. Western blot results showed that after overexpression of miR-138, the expression levels of PI3K, p-Akt, and p-mTOR in Tfh cells of patients with OS were distinctly reduced, and there was no obvious difference in the expression levels of Akt and mTOR. However, the ratio of p-Akt/Akt and p-mTOR/mTOR was dramatically lower, but the result turned to be opposite after inhibiting the miR-138 expression (Figures 3(a) and 3(b)). These results indicated that miR-138 can inhibit the activation of the PI3K/Akt/mTOR pathway in Tfh cells.

### 3.4. PDK1 Is Negatively Regulated by miR-138

We further studied the molecular mechanism of miR-138 regulating Tfh cell function. Through TargetScan (http://www.targetscan.org/vert_72/), we predicted that there was a binding site between miR-138 and PDK1, and the luciferase reporter experiment confirmed this suspect (Figure 4(a)). Subsequently, the mRNA and protein expression of PDK1 mRNA was upregulated in both OS patients and normal PBMC (Figures 4(b) and 4(c)). qRT-PCR was performed to detect the function of overexpressing miR-138 on PDK1 in Tfh cells of OS patients, and the results also showed that overexpression of miR-138 could inhibit the expression of PDK1 (Figure 4(d)), and its correlation analysis also represented that there was a negative correlation between miR-138 and PDK1 (Figure 4(e)), indicating that miR-138 can target and negatively regulate PDK1 in OS.

### 3.5. Influence of miR-138 on Tfh Cell Function Can Be Reversed by PDK1

The above results confirmed that miR-138 promoted the Tfh cell function and maturation of B cells, and miR-138 could target and negatively regulate PDK1. We further verified whether miR-138 regulated Tfh cells and B cells by changing PDK1. When miR-138 was overexpressed, the proportion of CD40L in CD4+CXCR5+ Tfh cells increased, and the ratios of p-Akt/Akt and p-mTOR/mTOR decreased dramatically. After coculturing, the positive rates of CD27 and CD38 in B cells became higher, while the secretion of IgM, IgG, IL-10, and IL-21 became more. However, the overexpression of PDK1 at the same time reversed the effect of miR-138 overexpression (Figures 5(a)–5(d)), suggesting that miR-138 can affect CD4+CXCR5+ Tfh cells by regulating PDK1, thereby further affecting the maturation of B cells.

## 4. Discussion

OS usually occurs in adolescents and children, mostly in their metaphysis of the long bones of the limbs, as well as other parts such as the ilium and spine [23–25]. It is a common primary malignant tumor with high incidence, rapid development, high degree of malignancy, and prone to metastasis, and its long-term survival rate is low [26]. Although surgery and neoadjuvant chemotherapy have made great progress, most patients still have a poor prognosis. In recent years, some scholars have also tried to apply gene therapies to OS, such as adenovirus-based gene transfection and siRNA-based gene silencing [27–29], and it has made some progress in some basic research at present.

The discovery of miRNA has brought scholars around the world to devote themselves to studying its role in tumors. At present, some miRNAs have been found that can promote or suppress cancer in tumors [30–32]. miR-138 is low expressed in a variety of malignant tumors and mainly suppresses cancer. In NSCLC, overexpression of miR-138 can inhibit the cell viability and invasion ability by directly targeting and negatively regulating FOXC1 [33]. Our previous finding shows that miR-138 is distinctly downregulated in human OS tissues and cell lines and suppresses the tumor suppressor [9]. In this study, it was also found that miR-138 was downregulated in OS tissue, which is consistent with previous findings. Immunotherapy for tumors has gradually become a research hotspot with its improving curative effect, and the immune microenvironment investigation is important in immunotherapy. Although miR-138 is known to suppress the tumor in OS [34], its function in the immune microenvironment of OS is not yet clear.

T cells are the most important cell group in the body's immune system. Tfh cells, a subgroup of CD4+ T cells with different functions, are a special type of helper T cells that may play an important role in the tumor microenvironment [35]. It differentiates in the germinal centers of secondary lymphoid organs and is an important regulator of antigen-specific B cell responses, which can promote the maturation of B cells and exert immune effects [36]. Studies have shown that in the microenvironment of chronic inflammatory breast cancer, the differentiation of human TFHX13 (tumor-infiltrating Tfh cells that produce CXCL13) cells may be a key factor in transforming Treg-mediated immunosuppression into adaptive antitumor humoral response de novo activation [37]. In this study, we also found that Tfh cells were notably higher in OS patients, and the expression of miR-138 was downregulated in Tfh cells. Overexpression of miR-138 can promote the expression of CD40L in Tfh cells, thereby promoting the maturation of B cells. All these studies showed that the activation of Tfh cells is essential in the immune microenvironment of tumor cells.

A study has shown that the PI3K-Akt-mTOR cascade is important in tumor cell proliferation, survival, angiogenesis, autophagy, and apoptosis [38], and it is also a common reason caused tumorigenesis and metastasis. According to the report, the PI3K/Akt cascade in OS is often overactivated to promote the occurrence, proliferation, and invasion of tumor cells [39]. Li et al. found that miR-122-5p regulated the activation of the PI3K-Akt-mTOR pathway by targeting the TP53 gene, inhibited OS cell proliferation, and promoted apoptosis [40]. In this study, we found that overexpression of miR-138 can notably inhibit the activation of the PI3K/Akt/mTOR pathway in Tfh cells, while interfering with miR-138 expression had the opposite result.

Phosphoinositide-dependent protein kinase 1 (PDK1) is an important regulator from the AGC protein kinase family, and it is also an essential protein in the PI3K/AKT pathway [41]. PDK1 plays a key role in cancer; in breast cancer, downregulating the PDK1 level can inhibit the migration and metastasis of breast cancer cells [42]. It has also been proved that in non-small-cell lung cancer, niR-145-3p can target PDK1 through the mTOR pathway to inhibit the invasion and migration of non-small-cell lung cancer cells [43]. miR-1271 can negatively regulate the AKT/mTOR pathway by targeting PDK1 to promote the apoptosis of pancreatic cancer cells [44]. However, there are few studies on miR-138 and PDK1 in OS Tfh cells. In this study, we found that miR-138 can directly target and negatively regulate PDK1 to inhibit the PI3K/Akt/mTOR pathway to regulate the immune microenvironment. At the same time, the reply experiment confirmed that PDK1 can reverse the effect of miR-138 on OS Tfh cells, suggesting that the miR-138/PDK1/PI3K/Akt/mTOR axis is expected to become a potential target for clinical treatment of OS.

## 5. Conclusion

To sum up, miR-138 inhibits the PI3K/Akt/mTOR pathway by targeting PDK1 to improve the ability of OS Tfh cells, thereby promoting the maturation of B cells and exerting immune function. This provides research guidance and a theoretical basis for the clinical treatment of OS.

## Figures and Tables

**Figure 1:** Expression of miR-138 in PBMCs and Tfh cells of OS patients. (a) miR-138 expression in serum PBMCs of patients with OS was detected by qRT-PCR; ^∗∗∗^*P* < 0.001. (b) Flow cytometry was performed to measure the proportion of CD4+CXCR5+ Tfh cells in CD4+ T cells in PBMCs. (c) Statistical map of the proportion of CD4+CXCR5+ Tfh cells. (d) Evaluation of the expression of miR-138 in CD4+CXCR5+ Tfh cells using qRT-PCR; ^∗∗^*P* < 0.01*vs.* the control group. (e) Correlation analysis between the expression of miR-138 and the proportion of CD4+CXCR5+ Tfh cells.

**Figure 2:** The function of miR-138 on B cell maturation in Tfh cells of patients with OS. (a) qRT-PCR verification of miR-138 expression in Tfh cells after interference or overexpression of miR-138. (b) Determination of the level of CD40L in Tfh cells of OS patients using flow cytometry. (c) The positive proportion changes of CD27 and CD38 in B cells after coculturing with CD4+CXCR5+ Tfh cells using flow cytometry detection. The level changes of (d) IgM, (e) IgG, (f) IL-10, and (g) IL-21 in the medium after coculturing with CD4+CXCR5+ Tfh cells using ELISA detection. ^∗^*P* < 0.05 and ^∗∗^*P* < 0.01*vs.* the NC mimics group; ^#^*P* < 0.05 and ^##^*P* < 0.01*vs.* the NC inhibitor group.

**Figure 3:** Effect of miR-138 on the PI3K/Akt/mTOR pathway in circulating Tfh cells in OS. (a) Evaluation of the expression levels of PI3K, Akt, p-Akt, mTOR, and p-mTOR in Tfh cells of patients with OS using Western blot. (b) Quantitative analysis results of protein expression levels. ^∗∗^*P* < 0.01*vs.* NC mimics; ^##^*P* < 0.01*vs.* NC inhibitor.

**Figure 4:** Targeting relationship between miR-138 and PDK1. (a) Verification of the binding site between miR-138 and using PDK1 dual-luciferase reporter gene experiment; ^∗∗^*P* < 0.01*vs.* the NC group. (b) Assessment of the expression of PDK1 in PBMC of patients with OS and normal people using qRT-PCR; ^∗∗∗^*P* < 0.001. (c) Determination of the expression of PDK1 in PBMC of patients with OS and normal persons using Western blot; ^∗∗^*P* < 0.01. (d) Evaluation of the expression of PDK1 in CD4+CXCR5+ Tfh cells of patients with OS using qRT-PCR; ^∗∗^*P* < 0.01*vs.* NC mimics; ^##^*P* < 0.01*vs.* NC inhibitor. (e) Correlation analysis of the relationship between miR-138 and PDK1 expression.

**Figure 5:** The role of PDK1 in the effect of miR-138 on Tfh cell function. (a) Changes of CD40L in each group of CD4+CXCR5+ Tfh cells using flow cytometry detection. (b) The positive rates and quantitative analysis results of CD27 and CD38 in B cells after coculturing with CD4+CXCR5+ Tfh cells using flow cytometry. (c) Assessment of changes in the levels of IgM, IgG, IL-10, and IL-21 in the cell culture after CD4+CXCR5+ Tfh cell coculturing with B cells using ELISA. (d) Determination of the expression levels and protein gray statistics of CD4+CXCR5+ Tfh cell PI3K, Akt, p-Akt, mTOR, and p-mTOR. ^∗∗^*P* < 0.01*vs.* NC mimics+NC vector; ^##^*P* < 0.01*vs.* miR-138+NC vector.

**Table 1:** Primer sequences.

Gene	Sequence (5′-3′)
miR-138	
Forward	GACCCAGATTCCACCATAT
Reverse	CAGTGCAGGGTCCGAGGT
U6	
Forward	UUCUCCGAACGUGUCACGUTT
Reverse	UGACACGUUCGGAGAATT
PDK1	
Forward	CTGTGATACGGATCAGAAACCG
Reverse	TCCACCAAACAATAAAGAGTGCT
GAPDH	
Forward	GGAGCGAGATCCCTCCAAAAT
Reverse	GGCTGTTGTCATACTTCTCATGG

## Data Availability

The data used to support the findings of this study are available from the corresponding author upon request.

## References

[1] Longhi A., Errani C., De Paolis M., Mercuri M., Bacci G. (2006). Primary bone osteosarcoma in the pediatric age: state of the art. *Cancer Treatment Reviews*.

[2] Seiter M., Al Maaieh M., Rosenberg A., Conway S. (2016). Primary osteosarcoma of the bone with rhabdoid features: a rare, previously undescribed primary malignant tumor of bone. *Case Reports in Surgery*.

[3] Sun R., Shen J., Gao Y. (2016). Overexpression of EZH2 is associated with the poor prognosis in osteosarcoma and function analysis indicates a therapeutic potential. *Oncotarget*.

[4] Felekkis K., Touvana E., Stefanou C., Deltas C. (2010). microRNAs: a newly described class of encoded molecules that play a role in health and disease. *Hippokratia*.

[5] Turchinovich A., Weiz L., Langheinz A., Burwinkel B. (2011). Characterization of extracellular circulating microRNA. *Nucleic Acids Research*.

[6] Pang L., Li B., Zheng B., Niu L., Ge L. (2017). miR-138 inhibits gastric cancer growth by suppressing SOX4. *Oncology Reports*.

[7] Wei Z. J., Liu J., Qin J. (2017). miR-138 suppressed the progression of osteoarthritis mainly through targeting p65. *European Review for Medical and Pharmacological Sciences*.

[8] Wang Z., Yao Y. J., Zheng F. (2017). Mir-138-5p acts as a tumor suppressor by targeting pyruvate dehydrogenase kinase 1 in human retinoblastoma. *European Review for Medical and Pharmacological Sciences*.

[9] Jiang B., Mu W., Wang J. (2016). MicroRNA-138 functions as a tumor suppressor in osteosarcoma by targeting differentiated embryonic chondrocyte gene 2. *Journal of Experimental & Clinical Cancer Research*.

[10] Roberto G. M., Lira R. C., Delsin L. E. (2020). microRNA-138-5p as a worse prognosis biomarker in pediatric, adolescent, and young adult osteosarcoma. *Pathology Oncology Research*.

[11] Wei J., Nduom E. K., Kong L. Y. (2016). MiR-138 exerts anti-glioma efficacy by targeting immune checkpoints. *Neuro-Oncology*.

[12] Li L., Lu S., Liang X. (2019). *γδ*TDEs: an efficient delivery system for miR-138 with anti-tumoral and immunostimulatory roles on oral squamous cell carcinoma. *Mol Ther Nucleic Acids*.

[13] Schaerli P., Willimann K., Lang A. B., Lipp M., Loetscher P., Moser B. (2000). CXC chemokine receptor 5 expression defines follicular homing T cells with B cell helper function. *The Journal of Experimental Medicine*.

[14] Liu X., Yan X., Zhong B. (2012). Bcl6 expression specifies the T follicular helper cell program in vivo. *Journal of Experimental Medicine*.

[15] Crotty S. (2014). T follicular helper cell differentiation, function, and roles in disease. *Immunity*.

[16] Guo Z., Liang H., Xu Y. (2017). The role of circulating T follicular helper cells and regulatory cells in non-small cell lung cancer patients. *Scandinavian Journal of Immunology*.

[17] Hollern D. P., Xu N., Thennavan A. (2019). B cells and T follicular helper cells mediate response to checkpoint inhibitors in high mutation burden mouse models of breast cancer. *Cell*.

[18] Gao W., Zhou J., Ji B. (2017). Evidence of interleukin 21 reduction in osteosarcoma patients due to PD-1/PD-L1-mediated suppression of follicular helper T cell functionality. *DNA and Cell Biology*.

[19] He L., Yang H., Huang J. (2021). The tumor immune microenvironment and immune-related signature predict the chemotherapy response in patients with osteosarcoma. *BMC Cancer*.

[20] Cumpelik A., Heja D., Hu Y. (2021). Dynamic regulation of B cell complement signaling is integral to germinal center responses. *Nature Immunology*.

[21] Wang F., Luo Y., Zhang L., Younis M., Yuan L. (2021). Down-regulation of LncRNA 2900052N01Rik inhibits LPS-induced B cell function _in vitro_. *Cellular Immunology*.

[22] Li J. B., Wang H. Y., Yao Y. (2017). Overexpression of microRNA-138 alleviates human coronary artery endothelial cell injury and inflammatory response by inhibiting the PI3K/Akt/eNOS pathway. *Journal of Cellular and Molecular Medicine*.

[23] Isakoff M. S., Bielack S. S., Meltzer P., Gorlick R. (2015). Osteosarcoma: current treatment and a collaborative pathway to success. *Journal of Clinical Oncology*.

[24] Anderson M. E. (2016). Update on survival in osteosarcoma. *The Orthopedic Clinics of North America*.

[25] Gianferante D. M., Mirabello L., Savage S. A. (2017). Germline and somatic genetics of osteosarcoma -- connecting aetiology, biology and therapy. *Nature Reviews. Endocrinology*.

[26] Ritter J., Bielack S. S. (2010). Osteosarcoma. *Annals of Oncology*.

[27] Rochette L., Lorin J., Zeller M. (2013). Nitric oxide synthase inhibition and oxidative stress in cardiovascular diseases: possible therapeutic targets?. *Pharmacology & Therapeutics*.

[28] Lin Y. H., Jewell B. E., Gingold J. (2017). Osteosarcoma: molecular pathogenesis and iPSC modeling. *Trends in Molecular Medicine*.

[29] Czarnecka A. M., Synoradzki K., Firlej W. (2020). Molecular biology of osteosarcoma. *Cancers*.

[30] Li Q., Li B., Li Q. (2018). Exosomal miR-21-5p derived from gastric cancer promotes peritoneal metastasis via mesothelial-to-mesenchymal transition. *Cell Death & Disease*.

[31] Wu M., Duan Q., Liu X. (2020). MiR-155-5p promotes oral cancer progression by targeting chromatin remodeling gene ARID2. *Biomedicine & Pharmacotherapy*.

[32] Yang Y., Bao Y., Yang G. K., Wan J., du L. J., Ma Z. H. (2019). MiR-214 sensitizes human colon cancer cells to 5-FU by targeting Hsp27. *Cellular & Molecular Biology Letters*.

[33] Bai X., Shao J., Zhou S. (2019). Inhibition of lung cancer growth and metastasis by DHA and its metabolite, RvD1, through miR-138-5p/FOXC1 pathway. *Journal of Experimental & Clinical Cancer Research*.

[34] Zhou Z., Li Z., Shen Y., Chen T. (2017). MicroRNA-138 directly targets TNFAIP8 and acts as a tumor suppressor in osteosarcoma. *Experimental and Therapeutic Medicine*.

[35] Sun Y., Zu J. C., Li H. F., Li Y. H., Li T. T. (2017). Research on follicular helper T cells (TFH) in tumor microenvironment. *Jiankang Qianyan*.

[36] Ma C. S., Deenick E. K., Batten M., Tangye S. G. (2012). The origins, function, and regulation of T follicular helper cells. *The Journal of Experimental Medicine*.

[37] Gu-Trantien C., Migliori E., Buisseret L. (2017). CXCL13-producing TFH cells link immune suppression and adaptive memory in human breast cancer. *JCI Insight*.

[38] Zhang J., Yu X. H., Yan Y. G., Wang C., Wang W. J. (2015). PI3K/Akt signaling in osteosarcoma. *Clinica Chimica Acta*.

[39] Xu Y., Li N., Xiang R., Sun P. (2014). Emerging roles of the p38 MAPK and PI3K/AKT/mTOR pathways in oncogene-induced senescence. *Trends in Biochemical Sciences*.

[40] Li K. W., Wang S. H., Wei X., Hou Y. Z., Li Z. H. (2020). Mechanism of miR-122-5p regulating the activation of PI3K-Akt-mTOR signaling pathway on the cell proliferation and apoptosis of osteosarcoma cells through targeting TP53 gene. *European Review for Medical and Pharmacological Sciences*.

[41] Gagliardi P. A., Puliafito A., Primo L. (2018). PDK1: at the crossroad of cancer signaling pathways. *Seminars in Cancer Biology*.

[42] Raimondi C., Falasca M. (2011). Targeting PDK1 in cancer. *Current Medicinal Chemistry*.

[43] Chen G. M., Zheng A. J., Cai J., Han P., Ji H. B., Wang L. L. (2018). microRNA-145-3p inhibits non-small cell lung cancer cell migration and invasion by targeting PDK1 via the mTOR signaling pathway. *Journal of Cellular Biochemistry*.

[44] Xie F., Huang Q., Liu C. H. (2018). MiR-1271 negatively regulates AKT/MTOR signaling and promotes apoptosis via targeting PDK1 in pancreatic cancer. *European Review for Medical and Pharmacological Sciences*.

